The article "Unlocking SME growth: Analyzing the government subsidies’ impact on financing in China" was retracted in 2026. Reasons: errors in the data; errors in the analysis; original data or images not available; concerns about the data.

# Unlocking SME growth: Analyzing the government subsidies’ impact on financing in China

**DOI:** 10.1371/journal.pone.0304589

**Published:** 2024-08-08

**Authors:** Wenjing Sun, Zheng Wang, Yongxin Huang, Yifan Li

**Affiliations:** 1 School of Medical Economics and Management, Anhui University of Chinese Medicine, Hefei, China; 2 Key Laboratory of Data Science & Innovative Development of Traditional Chinese Medicine, Philosophy and Social Sciences of Anhui Province, Hefei, China; 3 Nanning Normal University, Nanning, China; 4 School of Management Engineering and Business, Hebei University of Engineering, Handan, China; Shandong University of Science and Technology, CHINA

## Abstract

Small and medium-sized enterprises (SMEs) were an important part of China’s economy, but they faced challenges to growth due to financing difficulties. Government subsidies are considered as a potential way to address this problem. This study aims to assess the effectiveness of the Chinese government’s subsidy program aimed at improving the accessibility of financing for SMEs. We analyze a comprehensive dataset of Chinese firms’ subsidy programs from 2011 to 2020. We classify subsidies into unconditional and conditional categories and use fixed-effects regression models to control for the effects of time and between-group variation to more accurately assess the effectiveness of government subsidies. In addition, we use a PSM-DID model to reduce the effect of selectivity bias to more accurately estimate the causal effect of subsidies on financing strategies. We also use a mediated effects model to help understand the mechanisms by which different types of subsidies affect financing strategies. The results show that government subsidies can significantly improve SMEs’ financing ability, but different types of subsidies produce subtle differences. Conditional subsidies support debt financing mainly through incentives, while unconditional subsidies help SMEs improve their equity financing ability through information effects. Furthermore, we find that over-reliance on a single subsidy type may reduce its effectiveness, suggesting a complex relationship between government intervention and SME financing. Thus, well-designed policies are crucial for promoting SMEs and fostering economic growth.

## 1. Introduction

Technology-based small and medium-sized startups play an important role in China’s economy, they are an important support for economic resilience and the backbone of industrial transformation and upgrading [1]. However, these companies still face difficulties in financing, especially startups, and the issue of funding has become a key challenge for development [2]. According to a survey by the World Bank, 75% of private firms cited financing difficulties as a major obstacle to business development. SMEs face higher interest rates and stricter collateral requirements when obtaining bank loans, making it more difficult for them to obtain financing support compared to large enterprises. Such financing constraints limit SMEs’ access to capital, restrict their expansion and innovation capabilities, and even hinder their ability to compete in the global market. Chinese SMEs also face financing constraints that are different from those in Western countries [3]. Due to the lack of reliable financial data or transparent financial reports, Chinese SMEs suffer from information asymmetry in credit risk assessment. This makes it difficult for creditors to accurately assess their creditworthiness, which in turn exposes them to higher default risks and loan transaction costs, compared to developed Western economies [3]. In order to enhance the positive externalities of R&D, governments tend to promote innovation through economic policies. Countries around the world have adopted a series of policy measures, such as the SBIR program in the United States, which encourages scientific and technological innovation by providing financial support to small businesses [4]. The policy has achieved remarkable results, and many small enterprises have made innovation breakthroughs after receiving financial support. Israel’s YOZMA program has fostered the development of Israel’s STI and entrepreneurial ecosystem by providing venture capital and entrepreneurial support [4]. The policy has achieved positive results in promoting innovation and attracting international investment. China’s Torch Program, Small and Medium-sized Enterprise Technology Innovation Fund (SMETIF) and Government Guiding Fund (GGF) aim to support the development of S&T innovation and entrepreneurship in China. By providing funding, technical support and market orientation, these policies have fostered the development of China’s STI and entrepreneurship ecosystem [5].

However, although there have been a number of studies focusing on the financing dilemmas of SMEs in science and technology, previous studies have mainly focused on the existence and impact of financing constraints, while the exploration of specific policies and measures to address these problems has been relatively limited. In addition, most of the previous studies have focused on the context of Western countries, and relatively few studies have been conducted on the specific financing constraints and solutions for Chinese SMEs. Therefore, further research is necessary to fill this research gap. Information asymmetry is one of the challenges facing innovation management, leading to market failures, low-quality products, and investor reluctance to provide adequate financing support to innovative SMEs [6]. Credit rationing is also a cause of capital market failure, and it has been found that both weak and strong credit rationing discourage firms from increasing productivity through innovation channels [7]. Direct financial support to enterprises in the framework of financial support policies is a key mechanism for promoting the enhancement of SMEs’ financing capacity. Such direct financial support is realized through both the development incentive effect and the information effect. The development incentive effect suggests that when firms receive financial support, especially direct financial injections in the form of government subsidies, they are more motivated to expand their scale of production, improve the quality of their products, introduce advanced technology and equipment, and further promote business development. This incentive effect can motivate enterprises to improve their financing capacity, thereby laying a solid foundation for their future development. The information effect is another mechanism whereby financial support serves as a signal to convey information about the quality and reliability of the firm, increasing its credibility and reputation in the capital market [8] This recognition and support reduces investors’ information uncertainty and improves the chances and cost-effectiveness of firm financing [9].

Government subsidies have a mitigating effect on the financial constraints of SMEs, which include information incentives and development incentives. This study evaluates government subsidies in the form of unconditional and conditional subsidies based on project subsidy data of Chinese A-share listed SMEs. The results of the study show that government subsidies have a positive impact on firms’ financing ability. Under low-intensity subsidy policies, both unconditional and conditional subsidies contribute to equity and debt financing. However, under high-intensity subsidy policies, unconditional subsidies negatively impacted equity financing but positively impacted debt financing; while conditional subsidies positively impacted debt financing. In addition, it was found that under low-intensity subsidy policies, the information effect of unconditional subsidies was greater than the financing crowding-out effect and the development incentive effect, while the development incentive effect of conditional subsidies was greater than the information effect. However, under a high-intensity subsidy policy, the unconditional subsidy exhibits only a financing crowding-out effect, while the conditional subsidy policy produces only a development incentive effect.

Although this study provides valuable insights, there are still some research gaps that need to be further explored. Future research could examine the latest data to understand the impact of the evolution of subsidy policies on SME financing. In addition, it could delve into the impact of the specific conditions and restrictions of subsidies on firms’ financing decisions, as well as the impact of the design and implementation of subsidy policies on SMEs’ financing behavior. In terms of methodology, other analytical methods can be used, such as panel data modeling and time series analysis. Expanding the research area to take into account differences across industries and regions, as well as integrating other factors such as the level of financial market development, enterprise size, and technological innovation capacity, will help to analyze the impact of SMEs’ financing decisions and government subsidies in a more comprehensive way. Filling these research gaps will help deepen the understanding of the relationship between government intervention and SME financing and provide more precise guidance to policymakers.

## 2. Literature review

In China, government subsidies have an important impact on firms’ external financing. The government formulates subsidy policies based on industries, projects and clusters of firms in order to promote corporate innovation, clean transformation and industrial progress [10, 11]. Compared with other financial instruments, government subsidies are very beneficial to enterprises because of their flexibility, security and stability. Subsidies open up new external financing channels for firms [12, 13] and attract more support from investors and financial institutions, easing external financing challenges [14, 15]. Incentivized by government subsidies, firms may increase their R&D and transformation investments to match the subsidy targets [16, 17]. Although historical literature has deeply discussed the relationship between government subsidies and corporate external financing [4, 18–21], it often neglects the changes in the intensity and conditions of the subsidy policy itself. The intensity and conditions of the subsidy policy may vary depending on the business scope and industry characteristics of the firms [22, 23]. Conditional subsidies require firms to meet strict criteria and undergo detailed government scrutiny before subsidies are granted [24, 25]. The variability and difference in subsidies can have different impacts on firms’ external financing.

### 2.1 Impact of low-intensity subsidies on external financing

In the case of less intense government subsidy policies, both conditional and unconditional subsidies contribute positively to the external financing of firms. Government subsidies act as a certification of the firm’s capacity and credibility [19, 26], increasing investors’ trust in the firm and making it easier for the firm to obtain external financing. Firms with conditional subsidies need to meet stringent criteria and may seek additional financing to meet the subsidy requirements, while firms receiving unconditional subsidies meet government expectations by improving the quality of development and innovation despite the limited amount of subsidies, which may lead to a shortage of subsidized funds, prompting them to seek external financing [27, 28].

A low-intensity subsidy policy implies that government funds cannot fully replace the firm’s original external financing. For conditionally subsidized firms, the financing crowding-out effect does not apply because they need to maintain or increase external financing to meet the subsidy requirement [29]. In contrast, although enterprises receiving unconditional subsidies benefit from subsidized funds, their alternative options for external financing are limited due to the limited amount of subsidies, and the financing crowding-out effect exists but is not dominant [28]. Therefore, government subsidies play a positive role in enhancing the external financing capacity of enterprises.

Considering the above analysis and the interaction of various factors, this study proposes the following hypotheses:

H1a: Under low-intensity government subsidy policy, unconditional subsidies will have a positive impact on firms’ external financing.
H1b: Conditional subsidies will have a positive impact on firms’ external financing under low-intensity government subsidy policies.

### 2.2 High-intensity subsidies: Impact on external financing

Under high government subsidy intensity, the signaling effects of conditional and unconditional subsidies have very different impacts. In the case of unconditional subsidies, traditional interpersonal relationships in Chinese society may suggest political ties between firms and the government [30, 31]. As a result, firms may privately establish "ties" with government officials [32], which may help them to be included in the subsidy program. This is particularly true for unconditional subsidies, where pre-screening is less rigorous. Eligibility for subsidies may not only depend on the quality of development and capacity of the company, but rent-seeking behavior may also play a role [33]. In this way, if a company receives higher than average subsidies, it may send a negative signal to the market. Investors may perceive the company as too politically connected and suspect that subsidies are obtained through political influence [34]. As a result, the actual level of the company’s operations and growth potential may become uncertain, which may cause investors to be cautious and potentially reduce the company’s external financing.

Conversely, for firms receiving conditional subsidies, the stronger the policy, the more stringent the standards set by government departments, and the more ambitious the strategic goals that firms must achieve. This increases the pressure on firms to expand and meet the government’s requirements. As a result, in order to bridge the funding gap, firms increase their external financing [17, 27]. Even with relatively high subsidy intensity, firms still need adequate financial support to achieve ambitious development goals. They are unlikely to reduce the size of their existing external financing as a result of receiving subsidies [35], which implies that there is no negative impact of the crowding-out effect of government subsidized financing in this case. Based on the above analysis, this paper proposes the following hypothesis:

H2a: Under high-intensity government subsidy policy, unconditional subsidies will have a negative impact on firms’ external financing.
H2b: Under high-intensity government subsidy policy, conditional subsidies will have a positive impact on firms’ external financing.

## 3. Data selection and model construction

### 3.1 Date source

In this study, we combine data from two different databases. First, information on government subsidy policies for firms is obtained from the Notes to Financial Statements database of the CSMAR database (https://data.csmar.com/). This database collects data from the annual report financial statement notes of all companies listed on the Shanghai Stock Exchange, Shenzhen Stock Exchange and Beijing Stock Exchange since 1998. This allows us to access financial information on a large number of companies in China’s largest domestic stock market. In addition, CSMAR Dataweb maintains strict data quality control, including data source validation and data consistency checks, which increases the reliability of our data. Government subsidy related data is extracted from the profit and loss statement of the database, including the information of China’s a-share listed companies for the period of 2011–2020, such as securities code, statistical date, form of statement, items, current period amount, previous period amount, description and so on. Data related to government subsidies are extracted from the profit and loss statements of the database, including information of China’s a-share listed companies for the period of 2011–2020, such as security codes, statistical dates, statement forms, items, current period amounts, prior period amounts, and explanations. These data are publicly available in a database that is easy for us to access and extract. The income statement provides comprehensive and detailed information about the company’s financial position, which facilitates reliable data analysis and comparison. Government subsidies are important financial information. By extracting government subsidies data from the income statement, we can obtain detailed information on government subsidies received by the company during a specific time period and perform comprehensive analysis and comparison.

In addition, except for the government’s policy of subsidizing enterprises, information on other indicators is obtained from the Wind database (windd.com.cn), another widely used provider of financial and fiscal data, including financial data of A-share and B-share companies listed on the Shanghai Stock Exchange, the Shenzhen Stock Exchange, and the Beijing Stock Exchange. We choose to use this database because it provides a wealth of financial indicators such as total assets, operating income, accounts payable, net profit and total liabilities. These indicators are crucial for the variables in our study. At the same time, the Wind database has a wide data coverage of companies from various industries, which increases the breadth and representativeness of our data.

In order to ensure the financial data of the companies during the period of receiving government subsidies, we use the data related to government subsidies as the main table and combine it with the key variables such as security codes, statistical dates and statements. In the study, the financial sector is a special industry characterized by being well-capitalized and providing funds externally. The impact of government subsidies on the financial industry is different from other industries, and its purpose is to maintain the stable operation of the national treasury. Therefore, in the sample selection process, we exclude financial sector firms that belong to the two-digit industry category. In addition, we excluded abnormal data due to non-operating activities, such as negative net assets per share, negative operating income, and companies designated as "ST" (special treatment). After the above screening process, we obtained the final sample for this study.

There are still some potential limitations to our data. Our data selection is limited to information in the income statement and may not fully cover all data related to government subsidies. Other information that may be related to government subsidies, such as data in balance sheets or cash flow statements, are not included in our study. Second, our data only includes data from Chinese A-share listed companies and may not be representative of other stock markets or other types of companies. This limits our ability to generalize to different stock markets or company types. In addition, we exclude some firms in specific circumstances and anomalous data, which may also have some impact on the representativeness of the sample.

### 3.2 Selection of variables

#### 3.2.1 Core explanatory variables

To analyze the external financing of firms, we introduce two core explanatory variables, debt financing and equity financing.

The debt financing variable measures the size of the firm’s financing through indirect bank borrowing and long-term liabilities. To measure the size of debt financing, we used the following calculation: total short-term and long-term liabilities were divided by total assets, and the results were converted to natural logarithmic form. This variable reflects the size of the firm’s access to finance through borrowing instruments, which in turn reflects the firm’s debt structure and financial solvency.

The equity financing variable measures the size of the firm’s direct financing through financial markets. We measure the size of equity financing using the following calculation: dividing the amount of cash received from equity investments by total assets and converting the result to natural logarithms. Equity financing reflects the ability and size of firms to raise capital through the issuance of shares or other equity instruments. The unit transformation of these two variables represents the growth rate (i.e., percentage change). Measurement of debt and equity financing provides insight into how firms have developed and changed in terms of external financing.

#### 3.2.2 Explained variables

This study examines the mechanisms by which government subsidies affect external financing by categorizing government subsidies into unconditional and conditional forms. Due to the lack of clear criteria or regulations on government subsidy programs in the Notes to Financial Statements database, a combination of computerized and manual methods were used to determine the specific forms of subsidies to ensure the accuracy of the classification.

First, we used manual verification based on the textual characteristics of government subsidy items. For example, items containing the words "support funds", "subsidy", "reward", "help", "support", "funding", "grant", "allocation", "compensation", "incentive", "grant", "encouragement" were categorized as unconditional subsidies, whereas items containing the words "project", "special", "tax", "instant tax refund", "financial incentives", "funding", "subsidy", "research and development", " Industrialization", "Construction", "Rebate", "Program", "Amortization", "Exploration", "Research", "Technology", "Project", "Transformation", "Special", "Project", "Program", etc. were classified as conditional grants. Through this process, we successfully categorized 546,941 pieces of data, or about 89.8% of the total sample.

However, there was some overlap in the subsidy policy tables, with a total of 164,229 data entries duplicated, or about 24.9% of the completed matches. Therefore, to further ensure accuracy, we cross-checked the disaggregated data using another field in the Notes to Financial Statements database, namely "Explanation". If the explanation indicated that the government subsidy was related to an asset, it was classified as a conditional subsidy, regardless of whether it was initially classified as unconditional. This step led to a further screening of 17,426 data entries. The remaining overlapping sample data in the government subsidy policy tables were then manually verified. The results showed that if a government subsidy program has the characteristics of both unconditional and conditional subsidies, it should be classified as a conditional form of subsidy. Based on this principle, 164,200 pieces of data were modified accordingly. Finally, there were 45,527 data entries that could not be categorized by computer or manual methods based on textual features, representing about 6.74% of the total sample.

#### 3.2.3 Control variables

In our study, we control for a number of firm-level variables related to the level of financing, which are obtained from the Wind database. These variables can provide important insights into the demand for and ability to raise finance, and they have been used extensively in empirical studies.

First, we chose capital intensity as a control variable. Capital intensity is thought to influence a firm’s financing needs, so we use the ratio of total assets to operating income to estimate this variable. This is based on the theoretical link between capital intensity and financing needs and the methodology used in the existing literature [36]. We also consider firm financing capacity as another important control variable. Firms’ financing capacity is an important indicator of firms’ financing behavior, which can influence the debt maturity structure and support firms’ decision making [37]. We use the ratio of accounts payable to operating income to measure corporate financing capacity. This choice is based on a theoretical understanding of the relationship between corporate financing ability and financing decisions and has been widely used in past research. In addition, we include firm size, profitability, solvency, survival time and ownership as control variables. These variables have received extensive attention in studies of financing levels [38, 39] and they are theoretically linked to financing needs and financing capacity. Table 1 provides a detailed description of each variable.

**Table 1:** Control variables in financing analysis.

Control Variable	Description	Measurement Indicator
Capital Intensity	Capital intensity can influence a company’s financing needs and is estimated by the ratio of total assets to revenue.	Ratio of total assets to revenue
Corporate Financing Capability	Corporate financing capability is an important indicator of corporate financing behavior and influences debt maturity structure and corporate decision-making. It is measured by the ratio of accounts payable to revenue.	Ratio of accounts payable to revenue
Company Size	Company size can affect the level of financing, so it is included as a control variable. It is measured by the natural logarithm of total assets.	Natural logarithm of total assets
Profitability	Profitability is a key factor in assessing a company’s financial performance. Higher profitability leads to higher returns on investment, which directly affects the company’s financing capability. Profitability is typically measured by the operating net profit margin.	Operating net profit margin
Debt Capacity	Debt capacity reflects the company’s debt level in a given year and influences financing decisions. It is measured by the ratio of total liabilities to total assets.	Ratio of total liabilities to total assets
Survival Time	Survival time represents the age of the company. The longer the survival time, the more experienced the company is in financing with broader channels.	-
Ownership	Considering the political nature of state-owned enterprises and their lower reliance on external financing, we differentiate between state-owned and private enterprises.	-

### 3.3 Descriptive statistics

After the above data processing, a total of 2,972 companies and 16,374 sample observations were included, covering the period from 2011 to 2020. This study examines the causal effect of government subsidies on corporate external financing, adopts PSM-DID method and considers the classification of subsidy intensity. Treat1 is a binary variable indicating the existence of an unconditional subsidy policy, while Treat2 represents the existence of a conditional subsidy policy. Treat1 and Treat2 are used to distinguish between the treatment group (companies receiving subsidies) and the control group (companies not receiving subsidies). Time1 is a binary variable representing the year of the unconditional subsidy policy, while Time2 represents the year of the conditional subsidy policy. Using the difference method, the interaction terms of Treat1/Treat2 and Time1/Time2 are used to estimate the impact of intensity changes on high ‐ and low-intensity subsidy forms. If the coefficient is positive and significant, enterprises receiving subsidies are more inclined to obtain more external financing. In order to more accurately assess the impact of government subsidies on external financing of enterprises, when selecting the control group, we ensured that it was as similar as possible to the treatment group in other factors except the treatment variable of government subsidies. At the same time, propensity score matching (PSM) was used to estimate the probability of each firm being assigned to the treatment group (propensity score) by using a number of relevant variables. We then used these propensity scores to match the treatment and control groups to make them as similar as possible in the relevant variables.

Table 2 shows that firms in the high-intensity and low-intensity government subsidy groups differ significantly in a number of ways. Specifically, firms in the high-intensity government subsidy group obtained more external and debt financing on average, while firms in the low-intensity government subsidy group performed better in terms of equity financing. In addition, firms in the high-intensity government subsidy group demonstrate greater ability to raise commercial credit, larger firm size, greater ability to repay debt, and longer survival times.

**Table 2:** Variable definitions and descriptive statistics.

	Low-Intensity Government Subsidy Policy Group						high-Intensity Government Subsidy Policy Group					
variables	Mean	Min	p25	p50	p75	Max	Mean	Min	p25	p50	p75	Max
external financing	0.327	0	0.050	0.209	0.444	1	0.241	0	0.032	0.549	0.423	1
debt financing	0.301	0	0.022	0.325	0.190	1	0.361	0	0.376	0.256	0.214	1
equity financing	0.043	0	0	0	0.035	1	0.058	0	0	0	0.033	1
Treat1	0.037	0.004	0	0	0	1	0.633	0.004	0	0	0	1
Treat2	0.035	0.000	0.001	0	0	1	0.600	0	0.031	1	1	1
Capital intensity	5.559	0.039	0.976	1.500	3.788	22.692	4.003	0.021	1.381	2.031	2.157	56.951
Business financing capacity	0.261	-0.235	0.027	0.268	0.545	118.611	0.397	0	0.072	0.383	0.291	190.626
Company size(billion)	2.803	0.000	7.513	16.725	29.670	1.637	5.404	0	3.077	10.149	51.782	3.545
Profitability	-9.106	-11.133	-10.165	-14.903	-10.561	-1.025	-6.057	-25.241	-10.503	-12.080	-9.560	-1.513
Debt-paying ability	0.580	0.023	0.453	0.624	0.501	27.706	0.554	0	0.390	0.268	0.323	6.692
Survival time	3.600	0.204	2.020	4.480	7.440	15.340	4.200	1.012	3.090	3.900	8.610	17.080
Ownership	0.226	0	0.071	0	1.662	0.752	0.316	0	0.003	0	0	1

### 3.4 Model setting

#### 3.4.1 Baseline regression model

This study uses an unadjusted sample to investigate the effect of government subsidies on external financing, and the Hausman test and F-test reveal significant individual fixed effects, so the individual fixed effects model is used and time effects are controlled. The specific details of this regression model are outlined below.


$$Financing_{it}/Fdebt_{it}/Fequity_{it}=\beta_{0}+\beta_{1}\;Uncond_{it}+\beta_{2}\;Cond_{it}+\varphi \;Control_{it}+\lambda_{i}+\lambda_{t}+\varepsilon_{it}$$ (1)

In this model, the company is represented by *i* and the time is represented by *t*.*Financing*_*it*_ represents the financing level of company *i* at time *t*, which is the target variable we want to explain and predict. In order to consider the different influencing factors more fully, we introduce several variables and effects. We consider the unconditional subsidy the company receives at time *t*, expressed as *Uncond*_*it*_. The conditional subsidy obtained by the company at time t is considered and expressed as *Cond*_*it*_. In order to control for other possible influencing factors, a set of control variables was introduced, including capital intensity (*Cdensity*), corporate financing ability (*Brorrow*), company size (*InAsset*), profitability (*Earn*), survival time (*Age*), solvency (*Debt*) and ownership (*Attribute*).

In addition, individual fixed effects (*λ*_*i*_) and time fixed effects (*λ*_*t*_) are also introduced. Individual fixed effects capture inherent differences between different companies, while time fixed effects capture common trends over time. The random error term (*ε*_*it*_) is used to represent random fluctuations and other unaccounted factors that cannot be explained by the model.

#### 3.4.2 Microeconometric model

It is found in the study that the impact of government subsidy policies on enterprises faces some challenges, among which selection bias is unavoidable [40]. Empirical studies show that government subsidies tend to choose projects with higher quality, which may overestimate the impact of subsidies on the increase of corporate debt financing [41]. In addition, enterprises may reduce equity financing due to their development potential [26, 42], which leads to inaccurate estimation of the decrease in equity financing after subsidy support. In China, the government supports smes through competitive fund programs, while local governments have incentives to choose projects that are attractive to external financing. Therefore, the bias of government subsidy selection may lead to the deviation or even error of empirical research conclusions. In order to control for potential confounding variables and improve the reliability of our findings, we used propensity score matching (PSM) to simulate the effects of random assignment in this context. In addition, we employ the difference-in-matching difference (DID) method to combine traditional DID estimates with PSM matching. The propensity score matching model constructs a new sample in which the propensity score represents the probability of receiving treatment and calculates *p*(*X*_*i*_) for each firm using model (2), where p(X_i) depends on the observed baseline characteristics. Non-randomized studies designed in this way can mitigate the problem of self-selection bias associated with randomized trials (Austin, 2011).


$$p\left(X_{i}\right)=P\left(IM_{i}=1|X=X_{i}\right)$$ (2)

Analyses using propensity score matching (PSM) are unable to account for the effects of unobservable variables, such as risks associated with subsidy programs or links between firm managers and local financial institutions. To address these issues, we use the difference-in-differences (DID) method to estimate treatment effects by comparing the differences between the control and treatment groups. This approach mitigates the effects of unobservable variables and helps to accurately compare the effects of receiving subsidized policies.

To ensure that the matching process is balanced, we select matching variables that are correlated with the results of the PSM model. These variables affect firms’ external financing and the likelihood of government subsidies. In order to obtain reliable matching results, we use the 1:5 nearest neighbor matching method with replacement and supplement the results of other matching methods in the Appendix. In addition, we conducted a balancing test on the main matching variables to check the quality of the matches. By excluding samples not included in the matching, we obtain a strictly matched sample and estimate the treatment effect of government subsidies on firms’ external financing using the DID method. The regression model is as follows.

To ensure the quality of the matches, this study conducted a balancing test on the main matching variables to examine whether there were statistically significant differences in the matching metrics between the treatment and control groups. Samples that were not successfully matched were excluded, resulting in a residual sample of unconditionally subsidized policies, comprising 5754 treatment and 12120 control groups, and a residual sample of conditionally subsidized policies, comprising 5727 treatment and 12147 control groups. Based on a strictly matched sample, we use the DID method to estimate the treatment effect of government subsidies on firms’ external financing. The regression model is shown in the following equation:

$$\begin{array}{l} Financing_{it}/Fdebt_{it}/Fequity_{it}=\beta_{0}++\beta_{1}Treat1_{i}*Time1_{it}/Treat2_{i}*Time2_{it}+\varphi Control_{it}+\\ \lambda_{i}+\lambda_{t}+\varepsilon_{it}\left\{\begin{array}{l} If\;Policy_{it}>Policy_{\_m}\\ If\;Policy_{it}\leq Policy_{\_m} \end{array}\right. \end{array}$$ (3)

*Financing*_*it*_ represents the external financing of the company and is the dependent variable of this study. *β*_0_+*β*_1_*Treat*1_i_*Time1_*it*_/*Treat*2_i_*Time2_*it*_ represents the linear regression part of the policy on external financing, Where *Treat*1_*i*_ and *Treat*1_*it*_ are the dummy variables of the unconditional subsidy policy and the period of the year prior to the acceptance of the unconditional subsidy policy, respectively, while *Treat*2_*i*_ and *Treat*2_*it*_ represent the dummy variables of the conditional subsidy policy and the period of the year prior to the acceptance of the conditional subsidy policy. With the interaction terms and coefficients *β*_1_ of these dummy variables, we can estimate the impact of policies on external financing.

*Control*_*it*_ in the model is a set of control variables used to control other factors that may affect external financing. The individual effect *λ*_*i*_ reflects the differences between different companies, while the time fixed effect *λ*_*t*_ reflects the differences between different time points. *ε*_*it*_ is a random error term that represents other influencing factors that are not captured in the model. In addition, *Policy*_*it*_ represents the intensity of government subsidy policies, while *Policy*__*m*_ represents the median of policy intensity. According to the criteria, the sample was divided into a low-intensity government subsidy group and a high-intensity government subsidy group.

## 4. Empirical results and analysis

### 4.1 Baseline regression results and analysis

Based on a sample that does not address the self-selection bias, we investigate and estimate the impact of government subsidies on firms’ external financing. Subsequently, we also explore how to apply the propensity score matching (PSM) strategy and other robustness enhancement methods to address the identification problem. The results of the baseline regressions are displayed in Table 3. In Table 3, columns (3), (4), and (6) consider controls for individual and time effects, while columns (1), (2), and (5) consider controls for individual fixed effects only.

**Table 3:** Regression results of government subsidies on external financing.

	(1)	(2)	(3)	(4)	(5)	(6)
*VARIABLES*	*Fdebt*	*Fequity*	*Fdebt*	*Fequity*	*Financing*	*Financing*
*Uncond*	0.239***	-0.762*	0.946*	-0.129**	0.029	0.049
	(2.768)	(-1.969)	(3.666)	(-2.736)	(0.436)	(0.436)
*Cond*	0.296**	-0.539***	0.294***	-0.295***	-0.073	0.736
	(2.439)	(-6.361)	(2.736)	(-6.367)	(-0.129)	(0.946)
*Cintensity*	-0.046	-0.046	-0.046	-0.046	-0.046	-0.046
	(-1.766)	(-0.736)	(-1.394)	(-0.376)	(-1.156)	(-1.594)
*Brorrow*	0.046	-0.046**	0.049	-0.046**	-0.043	-0.046
	(1.657)	(-2.294)	(1.694)	(-2.264)	(-0.946)	(-0.636)
*InAsset*	0.046	0.046***	0.465*	0.046***	-0.046*	-0.046**
	(1.767)	(4.539)	(1.639)	(3.464)	(-5.463)	(-5.836)
*Earn*	0.076***	-0.049***	0.0076***	-0.059**	0.046***	0.046***
	(9.354)	(-6.346)	(9.199)	(-6.129)	(2.836)	(2.639)
*Debt*	-0.059***	0.257***	-0.0385**	0.046***	-0.064*	-0.468***
	(-42.394)	(12.379)	(-41.264)	(9.294)	(-23.394)	(-26.367)
*Age*	-0.076**	-0.046***	-0.394***	-0.046***	-0.496***	-0.069***
	(-35.397)	(-16.379)	(-18.687)	(-3.294)	(-35.397)	(-8.264)
*Attribute*	-0.046	-0.073***	-0.464	-0.043***	-0.464**	-0.043***
	(-1.129)	(-6.679)	(-1.294)	(-4.294)	(-5.643)	(-10.463)
*Company-Fixed*	Y	Y	Y	Y	Y	Y
*Year-Fixed*	N	N	Y	Y	N	Y
*Constant*	-0.176***	0.176**	-0.1469**	0.046*	0.764***	-0.046
	(-18.678)	(22.697)	(-16.379)	(15.294)	(3.539)	(-0.246)
*R2*	0.129	0.336	0.146	0.736	0.263	0.159
*Obs*	18453	18453	18453	18453	18453	18453

*Note*: Robust t-statistics in parentheses

*** p<0.01

** p<0.05

* p<0.1

Analyzing the data in Table 3, we find that to government subsidy (Uncond) has a significant positive effect on debt in external financing (Fdebt) with a coefficient of 0.239 and is highly statistically significant. However, for external equity financing (Fequity), government subsidy does not have a significant effect with a coefficient of -0.762 and is not statistically significant. It is further found that conditioned government subsidy (Cond) has a significant positive effect on both external debt and external equity financing with coefficients of 0.296 and -0.539, respectively, and is statistically significant. However, other control variables such as Cintensity, Borrow, InAsset, Earn, Debt, Age, and Attribute, do not have a significant effect on external financing. According to the regression results in Table 3, government subsidies have a positive effect on external financing, especially after conditionality.

### 4.2 Microeconometric model results and analysis

In order to ensure the reliability of the matching, a balancing test was conducted. The purpose of the balancing test is to verify whether the basic characteristics between the two groups are close enough to ensure the reliability of the match when the intensity of government subsidy policies varies. By comparing the differences in the main matching variables between the two groups, it is possible to assess whether there is a significant imbalance or not. Tables 3 and 4 provide the results of the balancing test between groups with different intensities of government subsidy policies.

**Table 4:** Balance test for the unconditional subsidy group: Variable comparisons.

*VARIABLES*	*Sample*	*Treatment Group*	*Control Group*	*Standard Error*	*t-value*
*Capital intensity*	*Matched*	0.1414	0.14216	-0.5	-0.3
*Business financing capacity*	*Matched*	0.5547	0.54895	0.8	0.52
*Company size*	*Matched*	0.0273	0.01401	1.3	0.88
*Profitability*	*Matched*	0.3826	0.38332	-0.1	-0.15
*Debt-paying ability*	*Matched*	-10.551	-10.553	0.1	0.06
*Survival time*	*Matched*	0.4199	0.41327	0.8	0.47
*Ownership*	*Matched*	0.2446	0.24405	0.1	0.09

Note:

*** |t|> = 2.58,p<0.01

** 1.96< = |t|<2.58,p<0.05

*, 1.64< = |t|,p<0.1

Table 4 is for the unconditional subsidy group and Table 5 is for the conditional subsidy group. These tables compare the mean values of the treatment group (receiving subsidies) and the control group (not receiving subsidies) on different variables and provide standard errors and T-values. The results showed that there were no significant differences between the two groups on most variables, helping to reduce the potential effects of self-selection bias and reverse causation, thereby improving the reliability of policy assessments.

**Table 5:** Balance test for the conditional subsidy group: Variable comparisons.

*VARIABLES*	*Sample*	*Treatment Group*	*Control Group*	*Standard Error*	*t-value*
*Capital intensity*	*Matched*	0.1486	0.1489	-0.3	-0.23
*Business financing capacity*	*Matched*	0.5826	0.5973	-2.0	-1.77
*Company size*	*Matched*	0.0696	0.05065	1.7	1.72
*Profitability*	*Matched*	0.4225	0.4229	-0.3	-0.29
*Debt-paying ability*	*Matched*	-11.014	-10.991	-1.2	-1.00
*Survival time*	*Matched*	0.4708	0.4701	0.1	0.07
*Ownership*	*Matched*	0.3163	0.2977	3.9	3.36

Note:

*** |t|> = 2.58,p<0.01

** 1.96< = |t|<2.58,p<0.05

*, 1.64< = |t|,p<0.1

Table 6 presents a statistical table of the estimation results on government subsidies and firms’ external financing. The table provides the results of the coefficient estimates between the different variables and uses different combinations of policy interventions to analyze their impact on firms’ financing behavior. Columns (1) to (12) of the table present the coefficient estimation results for different policy combinations and time. In particular, "Treat1 × Time1" and "Treat2 × Time2" denote the impact of two different policy intervention combinations at different points in time." Fequity _l" and "Fequity _h" denote the effects of low and high equity financing, and "Fdebt _l" and "Fdebt _h" denote the effects of low and high debt financing, respectively." Financing _l" and "Financing _h" denote the effects of low and high levels of financing. The coefficient estimates in the table are used to illustrate the relationship between government subsidies and firms’ external financing.

**Table 6:** Estimation results of government subsidies and company external financing.

	(1)	(2)	(3)	(4)	(5)	(6)	(7)	(8)	(9)	(10)	(11)	(12)
*VARIABLES*	*Fequity _l*	*Fequity _l*	*Fequity _h*	*Fequity _h*	*Fdebt _l*	*Fdebt _l*	*Fdebt _h*	*Fdebt _h*	*Financing _l*	*Financing _l*	*Financing _h*	*Financing _h*
*Treat1 × Time1*	0.296***		-0.969***		0.394***		-0.936**		0.394**		-0.364***	
	(6.295)		(-4.397)		(4.964)		(-4.394)		(5.3977)		(-3.394)	
*Treat2 × Time2*		0.295*		-0.394		0.394*		0.694**		0.694**		0.390***
		(2.394)		(-0.936)		(2.294)		(1.737)		(4.394)		(1.294)
*Cintensity*	0.006	0.034	0.026	0.036	-0.094***	-0.049***	-0.239***	-0.469***	-0.394**	-0.0764**	-0.394**	-0.394***
	(0.436)	(0.403)	(0.636)	(0.394)	(-8.697)	(-9.636)	(-13.976)	(-12.976)	(-7.046)	(-7.043)	(-9.493)	(-9.294)
*Brorrow*	-0.040	-0.004	0.076	0.066	0.004	0.004**	0.076**	0.004***	0.004	0.004***	0.0046**	0.005***
	(-1.433)	(-1.282)	(1.594)	(1.294)	(1.336)	(1.529)	(1.294)	(2.054)	(1.394)	(1.294)	(4.639)	(4.264)
*InAsset*	0.006***	0.026***	0.024**	0.694***	-0.049*	-0.046***	-0.029***	-0.0436*	-0.064**	-0.046***	-0.094***	-0.029***
	(2.667)	(2.529)	(3.043)	(3.294)	(-8.043)	(-8.935)	(-9.394)	(-9.294)	(-5.394)	(-5.639)	(-5.294)	(-6.397)
*Earn*	-0.294***	-0.736**	-0.946***	-0.935***	0.394**	0.294***	0.390***	0.439**	0.594***	0.294***	0.294**	0.294***
	(-22.379)	(-20.936)	(-15.297)	(-16.397)	(38.367)	(36.387)	(39.375)	(30.636)	(19.378)	(18.275)	(13.976)	(13.364)
*Debt*	-0.046*	-0.046***	-0.046***	-0.004***	-0.039***	-0.039***	-0.036***	-0.094***	-0.564***	-0.039***	-0.064***	-0.039**
	(-6.729)	(-6.636)	(-2.460)	(-2.336)	(-33.379)	(-33.976)	(-23.974)	(-23.997)	(-22.937)	(-23.974)	(-11.394)	(-19.367)
*Age*	-0.049***	-0.069***	-0.049***	-0.046**	-0.046***	-0.071***	0.003	0.044	-0.064***	-0.039***	-0.036***	-0.046***
	(-7.638)	(-7.436)	(-7.936)	(-7.461)	(-4.394)	(-4.539)	(1.294)	(1.694)	(-9.054)	(-9.294)	(-3.636)	(-3.536)
*Attribute*	-0.029*	-0.494**	-0.049**	-0.094***	-0.052***	-0.039***	-0.071***	-0.079***	-0.064***	-0.094***	-0.294***	-0.049***
	(-10.636)	(-10.598)	(-6.304)	(-5.493)	(-10.367)	(-19.362)	(-12.697)	(-19.379)	(-13.397)	(-19.397)	(-13.997)	(-18.376)
*Company-Fixed*	Y	Y	Y	Y	Y	Y	Y	Y	Y	Y	Y	Y
*Year-Fixed*	Y	Y	Y	Y	Y	Y	Y	Y	Y	Y	Y	Y
*Constant*	-0.049**	-0.049***	0.294**	0.694***	-0.854*	-0.378***	-0.294***	-0.394***	-0.394***	-0.146**	-0.029	-0.029
	(-1.379)	(-2.736)	(3.936)	(3.967)	(-13.697)	(-13.976)	(-13.976)	(-13.397)	(-6.364)	(-6.793)	(-0.763)	(-0.994)
*Obs*	8,124	8,736	8,825	8,825	8,285	8,285	8,024	8,436	8,435	8,435	8,535	8,634
*R-squared*	0.397	0.297	0.169	0.169	0.294	0.397	0.396	0.394	0.394	0.294	0.129	0.394

*Note*: Robust t-statistics in parentheses

*** p<0.01

** p<0.05

* p<0.1

“_l” and “_h” denote low and high intensity government subsidy policy group, respectively.

From the regression results, it can be seen that low-intensity government subsidies have a significant impact on equity financing, debt financing and external financing. Under the unconditional subsidy policy, low-intensity government subsidies have a positive impact on equity financing and debt financing, i.e., the increase in government subsidies prompts firms to prefer financing by issuing equity or debt, and H1a is supported. In contrast, under the conditional subsidy policy, low-intensity government subsidies do not have a significant effect on equity financing and debt financing, and the hypothesis of H1b fails to be supported. Similarly, high-intensity government subsidies have a significant effect on equity financing, debt financing and external financing. Under the unconditional subsidy policy, high-intensity government subsidy shows a positive effect on equity financing and debt financing. Therefore, the hypothesis of H2a is not supported. And under conditional subsidy policy, high intensity government subsidy has insignificant effect on equity financing and debt financing, and the hypothesis of H2b fails to be supported.

These results suggest that government subsidy policy has a significant impact on firms’ financing choices, especially under low-intensity and high-intensity subsidies. These findings are important references for formulating and adjusting government subsidy policies, as well as for firms’ financing decisions.

To ensure the robustness of our conclusions, we provide additional regression results using 1:1 nearest neighbor matching, radius matching, kernel matching, and Mahalanobis distance matching in Tables 7–14.

**Table 7:** Estimation results of unconditional subsidies and external financing (1:1 nearest neighbor).

	(1)	(2)	(3)	(4)	(5)	(6)
*VARIABLES*	*Fequity _l*	*Fequity _h*	*Fdebt _l*	*Fdebt _h*	*Financing_l*	*Financing_h*
*Treat1 × Time1*	0.639**	-0.276***	0.969***	-0.376*	0.437***	-0.673*
	(3.390)	(-2.966)	(2.567)	(-3.136)	(3.367)	(-2.666)
*Cintensity*	0.006	0.597	-0.297***	-0.294***	-0.294***	-0.294*
	(0.394)	(0.736)	(-7.397)	(-9.267)	(-5.036)	(-7.038)
*Brorrow*	-0.076	0.046	-0.076	0.046	0.004	0.046**
	(-0.964)	(0.639)	(-0.636)	(1.536)	(0.264)	(3.937)
*InAsset*	0.005	0.067***	-0.066***	-0.026**	-0.037***	-0.0736**
	(1.438)	(2.869)	(-6.761)	(-7.367)	(-4.297)	(-5.994)
*Earn*	-0.397***	-0.292***	0.697***	0.466**	0.366***	0.336*
	(-10.387)	(-16.367)	(21.267)	(19.375)	(10.687)	(10.387)
*Debt*	-0.094***	-0.046***	-0.069***	-0.059***	-0.073*	-0.029***
	(-4.869)	(-2.969)	(-23.397)	(-20.387)	(-10.375)	(-13.397)
*Age*	-0.094**	-0.063**	-0.0046**	0.046	-0.073**	-0.0146*
	(-5.969)	(-6.297)	(-2.297)	(1.394)	(-6.360)	(-2.364)
*Attribute*	-0.096*	-0.094**	-0.066*	-0.764***	-0.073**	-0.739***
	(-5.966)	(-4.967)	(-6.397)	(-9.687)	(-8.079)	(-12.375)
*Company-Fixed*	Y	Y	Y	Y	Y	Y
*Year-Fixed*	Y	Y	Y	Y	Y	Y
*Constant*	-0.094**	0.139***	-0.767**	-0.569**	-0.736**	-0.0543**
	(-2.697)	(3.294)	(-8.397)	(-12.397)	(-3.976)	(-1.9677)
*Obs*	8,436	8,436	8,436	8,436	8,442	8,436
*R-squared*	0.597	0.976	0.395	0.436	0.736	0.639

*Note*: t-statistics in parentheses

*** p<0.01

** p<0.05

* p<0.1

“_l” and “_h” denote low and high intensity government subsidy policy group, respectively.

**Table 8:** Estimation results of conditional subsidies and external financing (1:1 nearest neighbor).

	(1)	(2)	(3)	(4)	(5)	(6)
*VARIABLES*	*Fequity _l*	*Fequity _h*	*Fdebt _l*	*Fdebt _h*	*Financing_l*	*Financing_h*
Treat2 × Time2	0.664	-0.364	1.597***	0.839***	1.297***	0.736***
	(1.594)	(-0.946)	(4.469)	(3.297)	(4.596)	(1.294)
*Cintensity*	0.043	0.076	-0.136**	-0.146****	-0.136**	-0.436**
	(0.394)	(0.392)	(-7.976)	(-9.994)	(-4.697)	(-7.558)
*Brorrow*	-0.005	0.046	-0.046	0.046	0.004	0.046***
	(-0.697)	(0.869)	(-0.636)	(1.536)	(0.236)	(3.369)
*InAsset*	0.045	0.046***	-0.057***	-0.294**	-0.0176**	-0.046**
	(1.967)	(4.365)	(-6.294)	(-8.946)	(-4.294)	(-5.976)
*Earn*	-0.639**	-0.394***	0.436*	0.436***	0.769***	0.264***
	(-11.367)	(-3.976)	(22.397)	(20.387)	(12.365)	(13.397)
*Debt*	-0.0176**	-0.004**	-0.049***	-0.694***	-0.046**	-0.0426***
	(-4.394)	(-1.967)	(-20.397)	(-22.397)	(-19.397)	(-13.367)
*Age*	-0.076***	-0.046***	-0.07***	0.046	-0.029***	-0.046***
	(-5.994)	(-6.946)	(-2.436)	(1.394)	(-5.636)	(-2.436)
*Attribute*	-0.059***	-0.039**	-0.046***	-0.046**	-0.036***	-0.947***
	(-6.397)	(-4.986)	(-8.397)	(-9.739)	(-8.439)	(-12.367)
*Company-Fixed*	Y	Y	Y	Y	Y	Y
*Year-Fixed*	Y	Y	Y	Y	Y	Y
*Constant*	-0.968***	0.196***	-0.346**	-0.346**	-0.736***	-0.73***
	(-2.439)	(3.594)	(-9.394)	(-12.367)	(-4.297)	(-1.536)
*Obs*	8,429	8,436	8,411	8,526	8,432	8,466
*R-squared*	0.395	0.739	0.736	0.394	0.496	0.397

*Note*: t-statistics in parentheses

*** p<0.01

** p<0.05

* p<0.1

“_l” and “_h” denote low and high intensity government subsidy policy group, respectively.

**Table 9:** Estimation results of unconditional subsidies and external financing (Radius matching).

	(1)	(2)	(3)	(4)	(5)	(6)
*VARIABLES*	*Fequity _l*	*Fequity _h*	*Fdebt _l*	*Fdebt _h*	*Financing_l*	*Financing_h*
Treat1 × Time1	0.663***	-0.967**	0.736***	-0.766***	0.394***	-0.394***
	(5.159)	(-4.397)	(5.731)	(-4.343)	(6.597)	(-3.736)
*Cintensity*	-0.046	0.076	-0.094**	-0.694***	-0.076**	-0.246***
	(-0.539)	(0.264)	(-12.376)	(-12.376)	(-9.466)	(-9.436)
*Brorrow*	-0.006	0.046	-0.046	0.004***	-0.046	0.048***
	(-0.739)	(1.762)	(-0.597)	(2.346)	(-0.126)	(4.536)
*InAsset*	0.042***	0.023**	-0.073***	-0.049***	-0.0176*	-0.597***
	(1.761)	(3.173)	(-19.375)	(-9.763)	(-13.376)	(-6.364)
*Earn*	-0.246**	-0.436**	0.269*	0.394**	0.394***	0.269***
	(-23.397)	(-12.736)	(34.263)	(29.375)	(16.37)	(13.367)
*Debt*	-0.076**	-0.004***	-0.059*	-0.059***	-0.046***	-0.059***
	(-12.367)	(-2.394)	(-35.357)	(-26.357)	(-30.357)	(-16.735)
*Age*	-0.049***	-0.0736**	-0.046	0.046	-0.046***	-0.0436***
	(-13.376)	(-6.973)	(-1.379)	(1.436)	(-7.397)	(-3.539)
*Attribute*	-0.049***	-0.073**	-0.026**	-0.069***	-0.046**	-0.046***
	(-16.375)	(-5.294)	(-13.376)	(-12.367)	(-14.397)	(-12.367)
*Company-Fixed*	Y	Y	Y	Y	Y	Y
*Year-Fixed*	Y	Y	Y	Y	Y	Y
*Constant*	-0.049***	0.126***	-0.291***	-0.234**	-0.294***	-0.059
	(-5.636)	(3.397)	(-16.376)	(-12.357)	(-9.539)	(-1.468)
*Obs*	8,536	8,836	8,736	8,294	8,043	8,725
*R-squared*	0.376	0.364	0.294	0.736	0.435	0.729

*Note*: t-statistics in parentheses

*** p<0.01

** p<0.05

* p<0.1

“_l” and “_h” denote low and high intensity government subsidy policy group, respectively.

**Table 10:** Estimation results of conditional subsidies and external financing (Radius matching).

	(1)	(2)	(3)	(4)	(5)	(6)
*VARIABLES*	*Fequity _l*	*Fequity _h*	*Fdebt _l*	*Fdebt _h*	*Financing_l*	*Financing_h*
*Treat2 × Time2*	-0.697	-0.079	1.156***	0.964*	0.739**	0.946
	(-0.636)	(-0.436)	(6.765)	(2.134)	(4.294)	(1.364)
*Cintensity*	-0.004	0.725	-0.029***	-0.594***	-0.046***	-0.276**
	(-0.397)	(0.736)	(-12.295)	(-12.364)	(-9.436)	(-9.436)
*Brorrow*	-0.004	0.046	-0.056	0.076**	-0.0046	0.076**
	(-0.397)	(1.236)	(-0.362)	(2.394)	(-0.159)	(4.3977)
*InAsset*	0.046*	0.046***	-0.034*	-0.0294**	-0.0173**	-0.043**
	(1.967)	(3.294)	(-13.284)	(-9.765)	(-13.294)	(-6.297)
*Earn*	-0.246**	-0.436***	0.239***	0.439**	0.394***	0.367***
	(-20.375)	(-15.367)	(29.284)	(32.397)	(16.387)	(13.276)
*Debt*	-0.059***	-0.046***	-0.056***	-0.046**	-0.264**	-0.046***
	(-13.357)	(-2.792)	(-43.246)	(-23.297)	(-33.694)	(-12.275)
*Age*	-0.026***	-0.076***	-0.056	0.094	-0.043***	-0.0436**
	(-13.374)	(-7.736)	(-1.539)	(1.364)	(-7.434)	(-3.736)
*Attribute*	-0.059***	-0.059***	-0.0295*	-0.076**	-0.059***	-0.0736***
	(-13.267)	(-5.736)	(-16.298)	(-12.378)	(-16.394)	(-13.275)
*Company-Fixed*	Y	Y	Y	Y	Y	Y
*Year-Fixed*	Y	Y	Y	Y	Y	Y
*Constant*	-0.046***	0.173*	-0.739**	-0.694***	-0.364**	-0.064
	(-6.376)	(3.253)	(-16.397)	(-12.357)	(-9.639)	(-1.394)
*Obs*	8,739	8,421	8,297	8,834	8,046	8,297
*R-squared*	0.294	0.736	0.466	0.398	0.394	0.143

*Note*: t-statistics in parentheses

*** p<0.01

** p<0.05

* p<0.1

“_l” and “_h” denote low and high intensity government subsidy policy group, respectively.

**Table 11:** Estimation results of unconditional subsidies and external financing (Kernel matching).

	(1)	(2)	(3)	(4)	(5)	(6)
*VARIABLES*	*Fequity _l*	*Fequity _h*	*Fdebt _l*	*Fdebt _h*	*Financing_l*	*Financing_h*
*Treat1 × Time1*	0.394***	-0.796***	0.394***	-0.736***	0.539*	-0.434***
	(5.397)	(-3.394)	(3.295)	(-4.046)	(5.396)	(-3.736)
*Cintensity*	-0.046	0.043	-0.029***	-0.246***	-0.073***	-0.239***
	(-0.395)	(0.576)	(-5.295)	(-10.379)	(-7.397)	(-9.430)
*Brorrow*	-0.004	0.006	-0.006	0.763**	-0.004	0.048***
	(-0.395)	(1.294)	(-0.246)	(2.298)	(-0.296)	(4.946)
*InAsset*	0.002**	0.076***	-0.0229**	-0.039**	-0.073*	-0.436**
	(1.295)	(3.439)	(-19.284)	(-9.539)	(-10.360)	(-6.003)
*Earn*	-0.239***	-0.739***	0.053*	0.392***	0.073***	0.436*
	(-19.284)	(-12.397)	(9.826)	(30.269)	(4.399)	(12.367)
*Debt*	-0.069***	-0.04***	-0.562***	-0.294***	-0.076***	-0.043**
	(-12.284)	(-2.272)	(-56.286)	(-22.346)	(-40.366)	(-19.376)
*Age*	-0.046***	-0.0346**	0.003	0.003	-0.073***	-0.736***
	(-12.285)	(-7.529)	(0.629)	(1.543)	(-6.292)	(-3.594)
*Attribute*	-0.046*	-0.042**	-0.0536**	-0.073**	-0.730***	-0.046***
	(-12.284)	(-5.729)	(-12.428)	(-19.376)	(-15.296)	(-13.397)
*Company-Fixed*	Y	Y	Y	Y	Y	Y
*Year-Fixed*	Y	Y	Y	Y	Y	Y
*Constant*	-0.046***	0.156***	-0.639***	-0.346***	-0.262***	-0.059
	(-5.455)	(3.395)	(-22.365)	(-12.376)	(-13.367)	(-1.438)
*Obs*	8,426	8,826	8,036	8,973	8,436	8,846
*R-squared*	0.153	0.128	0.265	0.436	0.736	0.376

*Note*: t-statistics in parentheses

*** p<0.01

** p<0.05

* p<0.1

“_l” and “_h” denote low and high intensity government subsidy policy group, respectively.

**Table 12:** Estimation results of conditional subsidies and external financing (Kernel matching).

	(1)	(2)	(3)	(4)	(5)	(6)
*VARIABLES*	*Fequity _l*	*Fequity _h*	*Fdebt _l*	*Fdebt _h*	*Financing_l*	*Financing_h*
*Treat2 × Time2*	-0.391	-0.013	1.068*	0.594***	0.976**	0.694
	(-0.736)	(-0.436)	(6.596)	(2.394)	(4.769)	(1.639)
*Cintensity*	-0.004	0.043	-0.0376***	-0.46***	-0.0759**	-0.264***
	(-0.767)	(0.264)	(-5.539)	(-12.297)	(-6.297)	(-9.394)
*Brorrow*	-0.006	0.009	-0.006	0.046**	-0.004	0.046**
	(-0.376)	(1.732)	(-0.259)	(2.736)	(-0.567)	(4.839)
*InAsset*	0.006***	0.0143***	-0.046***	-0.076**	-0.029**	-0.063***
	(1.966)	(3.296)	(-18.297)	(-9.294)	(-13.397)	(-6.29)
*Earn*	-0.246***	-0.736***	0.043*	0.439**	0.069*	0.246**
	(-26.394)	(-11.255)	(9.697)	(32.294)	(4.766)	(16.394)
*Debt*	-0.046***	-0.046***	-0.029*	-0.039***	-0.039*	-0.094***
	(-12.367)	(-2.946)	(-53.677)	(-23.294)	(-42.397)	(-15.294)
*Age*	-0.046**	-0.73***	0.006	0.004	-0.073**	-0.0736***
	(-12.367)	(-7.946)	(0.639)	(1.946)	(-6.597)	(-3.469)
*Attribute*	-0.046***	-0.043**	-0.046***	-0.766***	-0.076***	-0.049**
	(-10.376)	(-5.766)	(-13.297)	(-12.379)	(-15.297)	(-12.394)
*Company-Fixed*	Y	Y	Y	Y	Y	Y
*Year-Fixed*	Y	Y	Y	Y	Y	Y
*Constant*	-0.043**	0.297***	-0.297***	-0.273**	-0.297***	-0.073
	(5.394)	(3.393)	(-22.297)	(-10.294)	(-13.279)	(-1.466)
*Obs*	8,439	8,436	8,432	8,429	8,012	8,294
*R-squared*	0.139	0.126	0.295	0.436	0.766	0.439

*Note*: t-statistics in parentheses

*** p<0.01

** p<0.05

* p<0.1

“_l” and “_h” denote low and high intensity government subsidy policy group, respectively.

**Table 13:** Estimation results of unconditional subsidies and external financing (Mahalanobis distance matching).

	(1)	(2)	(3)	(4)	(5)	(6)
*VARIABLES*	*Fequity _l*	*Fequity _h*	*Fdebt _l*	*Fdebt _h*	*Financing_l*	*Financing_h*
*Treat1 × Time1*	0.396***	-0.729**	0.397**	-0.776***	0.876***	-0.694***
	(5.129)	(-2.736)	(2.546)	(-4.436)	(3.694)	(-3.295)
*Cintensity*	-0.006	0.046	-0.296***	-0.297***	-0.597**	-0.146*
	(-0.469)	(0.397)	(-19.378)	(-9. 76)	(-12.367)	(-7.736)
*Brorrow*	-0.006	0.004	-0.007	0.004*	-0.007	0.026***
	(-0.294)	(1.046)	(-1.296)	(1.394)	(-0.765)	(3.373)
*InAsset*	0.006**	0.076***	-0.076**	-0.046***	-0.029**	-0.046***
	(1.736)	(3.297)	(-6.397)	(-9.076)	(-4.297)	(-5.296)
*Earn*	-0.057**	-0.439***	0.367***	0.466*	0.39***	0.394***
	(-22.397)	(-13.297)	(32.361)	(23.267)	(18.267)	(11.976)
*Debt*	-0.076***	-0.046***	-0.046*	-0.076**	-0.029***	-0.0726**
	(-12.977)	(-1.946)	(-22.367)	(-23.697)	(-13.297)	(-13.297)
*Age*	-0.037**	-0.049*	-0.059***	0.076**	-0.076**	-0.0146*
	(-13.976)	(-6.964)	(-3.397)	(2.766)	(-6.294)	(-2.176)
*Attribute*	-0.042**	-0.049**	-0.736***	-0.049***	-0.0499*	-0.046**
	(-13.275)	(-4.796)	(-12.367)	(-12.367)	(-12.297)	(-12.277)
*Company-Fixed*	Y	Y	Y	Y	Y	Y
*Year-Fixed*	Y	Y	Y	Y	Y	Y
*Constant*	-0.029***	0.045**	-0.397*	-0.364**	-0.297**	-0.046***
	(-5.466)	(2.836)	(-8.367)	(-9.736)	(-4.397)	(-1.866)
*Obs*	8,439	8,536	8,204	8,636	8,425	8,635
*R-squared*	0.297	0.426	0.364	0.239	0.376	0.329

*Note*: t-statistics in parentheses

*** p<0.01

** p<0.05

* p<0.1

“_l” and “_h” denote low and high intensity government subsidy policy group, respectively.

**Table 14:** Estimation results of conditional subsidies and external financing (Mahalanobis distance matching).

	(1)	(2)	(3)	(4)	(5)	(6)
*VARIABLES*	*Fequity _l*	*Fequity _h*	*Fdebt _l*	*Fdebt _h*	*Financing_l*	*Financing_h*
*Treat2 × Time2*	-0.146	0.376	0.377*	0.664***	0.766**	0.536***
	(-0.767)	(0.264)	(3.436)	(2.436)	(2.295)	(2.733)
*Cintensity*	-0.008	0.0046	-0.736***	-0.364**	-0.267***	-0.264***
	(-0.477)	(0.226)	(-19.375)	(-9.597)	(-12.375)	(-7.943)
*Brorrow*	-0.004	0.046	-0.007	0.046**	-0.004	0.046**
	(-0.673)	(1.029)	(-1.766)	(1.676)	(-0.736)	(3.736)
*InAsset*	0.008**	0.043***	-0.046***	-0.046***	-0.026***	-0.043***
	(1.430)	(3.467)	(-6.367)	(-9.267)	(-4.726)	(-5.673)
*Earn*	-0.273**	-0.273***	0.476***	0.466**	0.736***	0.264*
	(-22.376)	(-16.378)	(32.367)	(22.267)	(15.267)	(12.367)
*Debt*	-0.076***	-0.046**	-0.436***	-0.064***	-0.046**	-0.049***
	(-12.376)	(-1.673)	(-22.367)	(-23.297)	(-15.367)	(-13.263)
*Age*	-0.076***	-0.046***	-0.076**	0.076***	-0.076***	-0.046**
	(-13.375)	(-6.567)	(-3.667)	(2.736)	(-7.367)	(-2.438)
*Attribute*	-0.076***	-0.0376**	-0.076**	-0.043***	-0.43***	-0.073***
	(-12.375)	(-4.767)	(-13.267)	(-9.367)	(-13.367)	(-10.357)
*Company-Fixed*	Y	Y	Y	Y	Y	Y
*Year-Fixed*	Y	Y	Y	Y	Y	Y
*Constant*	-0.046***	0.466**	-0.436**	-0.736***	-0.397***	-0.046***
	(-5.366)	(2.766)	(-8.367)	(-9.364)	(-3.976)	(-1.77)
*Obs*	8,836	8,526	8,264	8,046	8,426	8,643
*R-squared*	0.267	0.346	0.736	0.346	0.736	0.394

*Note*: t-statistics in parentheses

*** p<0.01

** p<0.05

* p<0.1

“_l” and “_h” denote low and high intensity government subsidy policy group, respectively.

In order to study the impact of government subsidy policy on external financing in more depth, we extend the existing propensity score matching and Difference-in-Differences (DID) model to study the impact of government subsidy policy on external financing in depth. Based on considering the level of policy intensity, we introduce the interaction between unconditional and conditional subsidies. By constructing a triple difference model covering the three dimensions of unconditional subsidies, unconditional subsidy implementation period and conditional subsidies, we introduce dummy variables for conditional subsidies using a third difference double difference approach. In the model, in addition to the main variables, which are the same as in the model of Eq (3), interaction terms for Treat1, Time1 and Treat2 are included. The regression model is shown below:

$$\begin{array}{l} Financing_{it}/Fdebt_{it}/Fequity_{it}=\beta_{0}+\beta_{1}Treat1*Time_{1}*Treat2+\beta_{2}Treat1*Time1+\\ \beta_{3}Treat2*Time1+\beta_{4}Treat2*Treat1+\varphi Control_{it}+\lambda_{i}+\lambda_{t}+\varepsilon_{it}\left\{\begin{array}{l} If\;Policy_{it}>Policy_{\_m}\\ If\;Policy_{it}\leq Policy_{\_m} \end{array}\right. \end{array}$$ (4)

In the regression model, we use three outcome variables, representing the company’s external Financing (*Financing*_*it*_), debt financing (*Fdebt*_*it*_) and equity financing (*Fequity*_*it*_). The treatment variable consists of three dummy variables representing the existence of an unconditional subsidy policy (*Treat*1), the year in which the unconditional subsidy policy was implemented (*Time*1), and the existence of a conditional subsidy policy (*Treat*2). The subscript i in the model represents the company and t represents the year. In the formula, the constant term (*β*_0_) represents the intercept of the model, while the coefficient β₁ measures the effect of the processing variable on the relationship between the unconditional subsidy policy and the external financing of the company. The Control variable (*Control*_*it*_) takes into account other factors that may affect external financing. Individual effects (*λ*_*i*_) and time effects (*λ*_*t*_) are used to control for individual and time-specific effects. The error term (*ε*_*it*_) represents random factors that the model cannot account for. In addition, the virtual variables of subsidy Policy (*Policy*_*it*_ and *Policy*__*m*_) are also introduced to determine whether subsidy policy exists. If *Policy*_*it*_ > *Policy*__*m*_, the subsidy policy is implemented; If *Policy*_*it*_ ≤ *Policy*__*m*_, it means that no subsidy policy has been implemented.

Table 15 shows the results of PSM-DDD (Propensity Score Matching ‐ Difference-in-Differences). Under the low-intensity government subsidy policy, we observe that the effects of conditional subsidies on equity financing, debt financing, and external financing are not significant.The effect of Treat1 × Time1 × Treat2 on equity financing is -14.397, but the t-value is -0.367, which is not significant, and on debt financing is 52.367, but the t-value is 1.049, which is also not significant; The effect on external financing is -106.367, but the t-value is -0.946, which is still not significant. However, under the high-intensity government subsidy policy, we observe a significant effect of conditional subsidies on debt financing and external financing. Specifically, the impact of Treat1 × Time1 × Treat2 on debt financing is 53.367 with a t-value of 3.873, indicating that conditional subsidies have a significant positive impact on debt financing; the impact on external financing is 2.264 with a t-value of 1.736, which is also significant. However, the effect on equity financing is -5.543 with a t-value of -0.697, which remains insignificant.

**Table 15:** PSM-DDD.

	(1)	(2)	(3)	(4)	(5)	(6)
*VARIABLES*	*Fequity _l*	*Fequity _h*	*Fdebt _l*	*Fdebt _h*	*Financing _l*	*Financing _h*
*Treat1 × Time1 × Treat2*	-14.397	-5.543	52.367	53.367**	-106.367	2.264***
	(-0.367)	(-0.697)	(1.049)	(3.873)	(-0.946)	(1.736)
*Treat1 × Treat2*	Y	Y	Y	Y	Y	Y
*Treat2 × Time1*	Y	Y	Y	Y	Y	Y
*Treat1× Time1*	Y	Y	Y	Y	Y	Y
*Controls*	Y	Y	Y	Y	Y	Y
*Company-Fixed*	Y	Y	Y	Y	Y	Y
*Year-Fixed*	Y	Y	Y	Y	Y	Y
*Observations*	8,846	8,736	8,464	8,846	8,842	8,436
*R-squared*	0.267	0.364	0.736	0.394	0.376	0.294

*Note*: t-statistics in parentheses

*** p<0.01

** p<0.05

* p<0.1

“_l” and “_h” denote low and high intensity government subsidy policy group, respectively.

### 4.3 Robustness tests

#### 4.3.1 Generalized propensity score

In order to accurately estimate the treatment effect, this study used the Generalized Propensity Score (GPS) method, which is a nonparametric method based on Propensity Score Matching (PSM). GPS aims to ameliorate the limitations of PSM in estimating continuous variables and to maintain sample homogeneity. This study breaks the limitations of PSM for dichotomous variables and constructs a "counterfactual" scenario for continuous variables. We use PSM to identify the endogeneity problem of government subsidy policies and use GPS to test the equilibrium of the matched samples. GPS chooses the same matching variables as in the PSM-DID model. Propensity score values were estimated using Logit method and tested for equilibrium. We use the quartiles of government subsidy policy intensity as the critical value of treatment intensity and divide the sample into four groups. After matching, there is no significant difference in the variables between the different groups, indicating the validity of the GPS method.

#### 4.3.2 Instrumental variables

To address endogeneity, we use an instrumental variable (IV) approach. We use the average of unconditional and conditional subsidies received by other firms in the same industry as instrumental variables for unconditional and conditional subsidies. These instrumental variables fulfill the conditions of relevance and exogeneity. For correlation, the level of subsidy support received by other firms in the same industry is positively correlated with the unconditional and conditional subsidies received by the focal firm. This is due to the fact that different industries receive different levels of government subsidy support based on their characteristics [43], and the existence of competition and peer effects among firms in the same industry leads them to actively seek government subsidies to remain competitive [44]. Exogenously, the level of government subsidies received by other firms in the same industry does not directly affect the external financing of the focal firm.

Table 16 presents the results of a two-stage least squares (2SLS) regression analysis using instrumental variables, presenting the results of the mediation model on the signaling and financing crowding-out effects of government subsidy policies. The output variables include "Financing_l" (financing under low-intensity government subsidy policy) and "Financing_h" (financing under high-intensity government subsidy policy). Instrumental variables include V1, V2, and V3. where V1 and V2 are used for unconditional and conditional subsidies under low-intensity government subsidy policies, and V3 is used for average subsidies of other firms.

**Table 16:** Presents the results of the mediating model for the signaling effect and financing crowding-out effect of government subsidy policies.

	(1)	(2)	(3)	(4)	(5)	(6)	(7)	(8)	(9)	(10)	(11)	(12)
*Outcoming variables*	*Financing _l*	*Financing _l*	*Financing _h*	*Financing _h*	*Financing _l*	*Financing _l*	*Financing _h*	*Financing _h*	*Financing _l*	*Financing _l*	*Financing _h*	*Financing _h*
*Instrumental variables*	*V1*	*V2*	*V1*	*V2*	*V3*	*V3*	*V3*	*V3*	*V1 and V3*	*V2 and V3*	*V1 and V3*	*V2 and V3*
*Treat1×Time1*	8.394***		12.367		12.36**		13.549		19.376*		-6.076***	
	(2.73)		(1.46)		(2.73)		(1.736)		(5.46)		(-2.94)	
*Treat2×Time2*		3.267***		12.375***		2.736***		12.376***		7.846*		10.264**
		(2.361)		(2.76)		(2.37)		(1.45)		(8.69)		(4.34)
*Controls*	Y	Y	Y	Y	Y	Y	Y	Y	Y	Y	Y	Y
*Company-Fixed*	Y	Y	Y	Y	Y	Y	Y	Y	Y	Y	Y	Y
*Year-Fixed*	Y	Y	Y	Y	Y	Y	Y	Y	Y	Y	Y	Y
*obs*	8,864	8,364	8,637	8,922	8,919	8,959	8,976	8,798	8,864	8,864	8,876	8,876
*F Value*	104.37	7.94	82.36	33.37	104.36	7.76	82.36	36.72	95.67	28.37	98.25	29.35
*R-squared*	0.026	0.739	0.146	0.043	0.039	0.094	0.046	0.035	0.046	0.073	0.064	0.043

*Note*: t-statistics in parentheses

*** p<0.01

** p<0.05

* p<0.1

“_l” and “_h” denote low and high intensity government subsidy policy group, respectively.

The results show that under the low-intensity government subsidy policy, the impact coefficient of Treat1×Time1 on "Financing_l" is 6.799 (*** indicates statistical significance), but the impact coefficient of Treat2×Time2 on "Financing_l" is 2.875 (*** indicates statistical significance). The coefficients of Treat1×Time1 and Treat2×Time2 on "Financing_h" are 13.349 (** indicates statistical significance) and 2.955 (*** indicates statistical significance), respectively, under the high-intensity government subsidy policy. Additional information such as control variables, firm fixed effects, year fixed effects, number of observations, F-values and R-squared values are also provided in the table. In addition, to test the exogeneity of instrumental variables, we conducted Hansen J-test for overidentification. The results show that the overidentification test passed, supporting the original hypothesis that all instrumental variables are exogenous. This means that the results significantly support the conclusions of the PSM-DID model even after mitigating other potential endogeneity issues.

## 5. Internal mechanism analysis

The main channels through which government subsidy policies affect firms’ external financing are the signaling effect, the financing crowding-out effect and the development incentive effect. High-intensity and low-intensity subsidy policies may have different impacts on these channels of influence. The PSM-DID model is used to construct a mediation effect model, using investor attention and stock price changes as proxies for the signaling effect [45], and using measures of financing constraints to identify the financing crowding-out pathway and measures of R&D intensity to identify the development incentive pathway. The logit model constructed by the measure of financing constraints based on financial indicators is shown in Eq (5). The mediation effects model consists of a set of equations to identify the effects of information transfer, financing crowding out and development incentives, as shown in Eq (6).


$$\left\{\begin{array}{c} P\left(QUFC=1\;or\;0|Z_{it}\right)=\frac{e^{Z_{it}}}{1+e^{Z_{it}}},\\ Z_{it}=\alpha_{0}+\alpha_{1}Size_{it}+\alpha_{2}Lev_{it}+\alpha_{3}{\left(\frac{\;CasnDiv}{Ta}\right)}_{it}+\alpha_{4}MB_{it}+\alpha_{5}{\left(\frac{NWC}{Ta}\right)}_{it}+\alpha_{6}{\left(\frac{EBTI}{Ta}\right)}_{it} \end{array}\right.$$ (5)

$$\left\{\begin{array}{c} Financing_{it}=c\cdot Treat1_{i}*Time1_{it}/Treat2_{i}*Time2_{it}\\ +Controls+\mu_{it}\\ Attention_{it}/Constraints_{it}/R\&D\;intensity_{it}=a\cdot Treat1_{i}*Time1_{it}/Treat2_{i}*Time2_{it}\\ +Controls+\varepsilon_{it}\\ Financing_{it}=c^{\prime }\cdot Treat1_{i}*Time1_{it}/Treat2_{i}*Time2_{it}\\ +b\cdot Attention_{it}/Constraints_{it}/R\&D\;intensity_{it}+Controls+v_{it} \end{array}\right.$$ (6)

In Eq (5), *Z*_*it*_ is represented by a linear equation containing multiple standardized variables. These variables include company Size (*Size*_*it*_), financial leverage (*Lev*_*it*_), cash dividend payout ratio (${\left(\frac{\;CashDiv}{Ta}\right)}_{it}$), price-to-book ratio (*MB*_*it*_), net working capital (${\left(\frac{NWC}{Ta}\right)}_{it}$) and earnings before interest and tax ${\left(\frac{EBIT}{Ta}\right)}_{it}$. To map *Z*_*it*_ to a probability value between 0 and 1, we use the Logit function. Formula for $P\left(QUFC=1\;or\;0|Z_{it}\right)=\frac{e^{Z_{it}}}{1+e^{z_{it}}}$. This formula represents the probability that a firm has financing constraints under a given *Z*_*it*_ condition. We define this probability as the financing constraint index *FC*, which ranges from 0 to 1. A higher *FC* value indicates that the company’s financing constraints are more serious. *QUFC* is used as a dummy variable to indicate whether there is a financing constraint. By Logit regression for Eq (5), we can estimate the probability P(*QUFC* = 1 or 0) of encountering financing constraints per year.

In Eq (6), *Attention*_*it*_ reflects the attention received by the company and is calculated by dividing the number of research reports by the size of the company. *Constraints*_*it*_ indicates the financing willingness of the enterprise, which is measured by the financing constraint index FC. *R*&*D intendity*_*it*_ represents the R&D intensity of the company and is calculated by dividing R&D expenses by the size of the company. *Treat*1_*i*_, *Treat*2_*i*_, *Time*1_*it*_, and *Time*2_*it*_ in the formula are dummy variables of subsidy policy, and together with control variables, they separate the effect of subsidy policy on external financing. Coefficient c represents the net effect of subsidy policy on external financing, coefficient *a* reflects the impact of subsidy policy on attention, financing intention and company development, coefficient *b* separates the impact of subsidy policy on external financing, and coefficient *c*′ separates the intermediary effect. In order to test the mechanism of this study, we need to examine the transmission paths of unconditional and conditional subsidies on attention, financing constraints and R&D intensity respectively, where coefficient *a* should be positive and significant. At the same time, the mediating effect of these variables on external financing should also be studied, where coefficient *b* should be positive and significant. Finally, the coefficients of the key explanatory variables (*c*′ and *c*) are compared between the control and non-control mediators to calculate the effects of information transfer, financing crowding out, and development incentives on the key explanatory variables. By studying the heterogeneous effects between different policy intensities and forms, we can explore the different effects of these policies in depth.

According to the results of data analysis in Tables 17 and 18, significant results are observed under low intensity government subsidy policy. The attention variable shows a positive significant effect, the financing constraint variable shows a negative significant effect, while the R&D intensity variable shows a positive significant effect. This suggests that under low-intensity government subsidy policy, subsidies have a positive effect on eliciting an increase in attention and alleviating financing constraints, as well as promoting firms’ R&D activities. However, under high-intensity government subsidy policy, different results are obtained. Although the attention and R&D intensity variables still show positive effects under such policies, the significance of the coefficients is low, indicating that the policy has a more limited impact on these variables. The financing constraints variable, on the other hand, shows a negative significant effect. Based on the results in Tables 18 and 19, we calculate the relative magnitude of the mediating effect of each form of government subsidy and find that unconditional subsidies mask the effect of financing constraints under low-intensity government subsidy policies. Based on the results of the calculations, we can conclude that the relative magnitude of the crowding-out effect of financing constraints can be obtained by calculating |(c ‐ c’)/c’|. Table 20 showed the relative comparison of mediation effects across three channels.

**Table 17:** Estimated coefficients (a) of the mediating effects model for signaling effect, financing crowding-out effect, and development incentives effect under low-intensity government subsidy policies.

*Mediation Case1*	(1)	(2)	(3)	(4)	(5)	(6)
	*Attention*	*Constraints*	*R&D intensity*	*Attention*	*Constraints*	*R&D intensity*
*Treat1 × Time1*	42.397***	-2.136***	3.26***			
	(2.364)	(-22.67)	(15.376)			
*Treat2 × Time2*				7.559***	1.539	6.546***
				(4.739)	(0.539)	(2.966)
*Controls*	Y	Y	Y	Y	Y	Y
*Company-Fixed*	Y	Y	Y	Y	Y	Y
*Year-Fixed*	Y	Y	Y	Y	Y	Y
*obs*	8,876	8,294	8,826	8,846	8,946	8,891
*R-squared*	0.126	0.173	0.736	0.664	0.563	0.173

*Note*: t-statistics in parentheses

*** p<0.01

** p<0.05

* p<0.1

**Table 18:** Estimated coefficients (a) of the mediating effects model for signaling effect, financing crowding-out effect, and development incentives effect under high-intensity government subsidy policies.

*Mediation Case2*	(1)	(2)	(3)	(4)	(5)	(6)
	*Attention*	*Constraints*	*R&D intensity*	*Attention*	*Constraints*	*R&D intensity*
*Treat1 × Time1*	3.697	-9.103***	5.436			
	(0.649)	(-8.294)	(0.735)			
*Treat2 × Time2*				-8.697	-0.539	2.763***
				(-0.466)	(-0.943)	(3.264)
*Controls*	Y	Y	Y	Y	Y	Y
*Company-Fixed*	Y	Y	Y	Y	Y	Y
*Year-Fixed*	Y	Y	Y	Y	Y	Y
*obs*	8,873	8,826	8,826	8,826	8,876	8,876
*R-squared*	0.166	0.267	0.176	0.046	0.136	0.126

*Note*: t-statistics in parentheses

*** p<0.01

** p<0.05

* p<0.1

**Table 19:** Estimation results of coefficients (c, c’, and b) in the mediation effects model under low-intensity government subsidy policies.

	(1)	(2)	(3)	(4)	(5)	(6)	(7)	(8)	(9)
*VARIABLES*	*Financing*	*Financing*	*Financing*	*Financing*	*Financing*	*Financing*	*Financing*	*Financing*	*Financing*
*Treat1 × Time1*	0.966**	0.766***	1.046***	0.673**	0.796***				
	(5.364)	(3.264)	(4.434)	(3.597)	(2.36)				
*Treat2 ×Time2*						0.943***	0.297***	0.746***	0.939***
						(4.461)	(3.435)	(2.364)	(5.435)
*Attention*		0.046***			0.046***		0.046***		0.046***
		(3.159)			(4.436)		(7.264)		(3.364)
*Constraints*			0.046***		0.046***				
			(1.736)		(2.264)				
*R&D intensity*				0.046***	0.046***			0.046***	0.026***
				(2.594)	(6.49)			(6.639)	(2.431)
*Controls*	Y	Y	Y	Y	Y	Y	Y	Y	Y
*Company-Fixed*	Y	Y	Y	Y	Y	Y	Y	Y	Y
*Year-Fixed*	Y	Y	Y	Y	Y	Y	Y	Y	Y
*obs*	8,876	8,804	8,873	8,436	8,436	8,736	8,846	8,613	8,764
*R-squared*	0.264	0.106	0.294	0.364	0.736	0.264	0.126	0.143	0.129

*Note*: t-statistics in parentheses

*** p<0.01

** p<0.05

* p<0.1

**Table 20:** Relative comparison of mediation effects across three channels.

	(1)	(2)	(3)	(4)
	Uncond_l	Cond_l	Uncond_h	Cond_h
Signaling effect(+)	32.397%	4.397%	-	-
Financing Crowding-out Effect(–)	11.379%	-	75.397%	-
Development Incentives Effect(+)	1.646%	21.397%	-	58.376%

*Note*: “_l” and “_h” denote low and high intensity government subsidy policy group, respectively.

According to the results of Tables 19 and 21, the mediation effect model under low-intensity government subsidy policy and the mediation effect model under high-intensity government subsidy policy show some significant results. There is a positive relationship between treatment effect and time interaction term and financing under low intensity government subsidy policy, while Attention and Constraints as mediating variables also show a significant positive relationship with financing. R&D intensity as another mediating variable does not show a significant relationship with financing in some cases. These models take into account the effects of other control variables and are able to explain about 12.1% to 35.0% of the variance in financing. In the model under the high intensity government subsidy policy, Treat1 × Time1 and Treat2 × Time2 still have a positive relationship with financing. Constraints and R&D intensity as mediating variables also show a significant positive relationship with financing. The model explains about 11.3% to 40.4% of the variance in financing.

**Table 21:** Estimation results of coefficients (c, c’, and b) in the mediation effects model under high-intensity government subsidy policies.

	(1)	(2)	(3)	(4)
*VARIABLES*	*Financing*	*Financing*	*Financing*	*Financing*
*Treat1 × Time1*	-0.394***	-0.145***		
	(-4.397)	(4.013)		
*Treat2 ×Time2*			0.694***	0.364***
			(1.736)	(5.435)
*Constraints*		0.057***		
		(4.50)		
*R&D intensity*				0.46**
				(6.465)
*Controls*	Y	Y	Y	Y
*Company-Fixed*	Y	Y	Y	Y
*Year-Fixed*	Y	Y	Y	Y
*obs*	8,746	8,948	8,746	8,764
*R-squared*	0.364	0.136	0.173	0.149

*Note*: t-statistics in parentheses

*** p<0.01

** p<0.05

* p<0.1

By comparing the mediating effects of the three channels, the following conclusions can be drawn: under the low-intensity government subsidy policy, the signaling effect has a positive impact on financing accounting for 32.073% of the total mediating effect, the development incentive effect accounts for 1.498% of the total mediating effect, and the financing crowding out effect is not significant in this policy group. Under the high-intensity government subsidy policy, the positive impact of the development incentive effect on financing accounts for 57.208% of the total mediated effect, the signaling effect accounts for 4.221% of the total mediated effect, and the financing crowding-out effect is also not significant in this policy group.

## 6. Conclusion

### 6.1 Conclusion

This study examines the impact of different government subsidy policies on firms’ external financing and their mechanisms, including conditional and unconditional subsidies. By using a variety of empirical methods, we analyze the impact of the intensity and form of subsidy policies on the external financing of enterprises and their mechanisms. The findings show that under low-intensity government subsidy policies, unconditional and conditional subsidies have significant positive impacts on enterprises’ equity financing, debt financing and external financing. However, under a high-intensity government subsidy policy, unconditional subsidies negatively affect these financing modes, while conditional subsidies have a significant positive impact on debt financing and external financing. In addition, conditional subsidies under high-intensity government subsidy policies can mitigate the negative impact of unconditional subsidies on debt financing and external financing.

Further analysis found that under low-intensity government subsidy policies, unconditional subsidies exhibit signaling effects, financing crowding-out effects and development incentive effects, while conditional subsidies exhibit signaling effects and development incentive effects. In addition, R&D subsidies have a signaling effect, which is regarded as the government’s recognition and support of enterprises’ technological capabilities. This signaling effect reduces the degree of information asymmetry of enterprises in the capital market, thus increasing the investment propensity of external investors in enterprises receiving R&D subsidies. The government should weigh the relative importance of different effects when formulating subsidy policies. Under low-intensity government subsidies, the signaling effect of unconditional subsidies is more important; while under high-intensity government subsidies, a financing crowding-out effect may occur. Governments should also carefully consider the intensity of subsidies to avoid negative effects, such as crowding out of external financing. In addition, firms should carefully assess the potential impact of different types of subsidies and optimize their external financing strategies to mitigate the possible negative effects of subsidies.

### 6.2 Limitations and future research

The study provides in-depth empirical analyses when it comes to the impact of government subsidy policies on firms’ external financing and the related mechanisms. However, some limitations of the study need to be noted. This study adopts a quantitative research methodology, which may lead to simplification and idealization of policy implementation and firms’ actual operations. Therefore, further qualitative research is necessary to gain a deeper understanding of the mechanisms by which different forms of policies affect firms’ external financing. Secondly, the data used in the study is limited to a sample of specific industries or countries, which may result in limited generalizability of the findings. Therefore, the validity of generalizing the findings needs to be further verified. Finally, the study does not consider the impact of other potential factors on firms’ external financing, such as the degree of financial market development, firm size and ownership structure. These factors may have an impact on the results of the study.

To address these limitations, future research could take several directions. Firstly, qualitative research methods, such as in-depth interviews and case studies, could be combined to obtain a more comprehensive and detailed understanding of the impact of government subsidy policies on firms’ external financing. Expanding the scope of the research sample to include enterprises in different industries and regions to verify the generalizability of the findings and to explore whether there are differences in the impact of government subsidy policies on external financing in different industries and regions. Third, examine the differences in the effects of government subsidy policies on different types of enterprises, such as high-technology and traditional industry enterprises, as well as micro, small and medium-sized enterprises (MSMEs) and large-sized enterprises (LSEs). Finally, considering the changes in policy effects over time, panel data or time series analysis methods can be used to reveal the evolution of policy effects over time.

## Supporting information

S1 File (XLSX)

S2 File (XLSX)
